The article "Effect of Eye Movement Training on Sleep Quality of Patients with Advanced Lung Cancer Based on Pittsburgh Sleep Quality Index" was published in 2021. Journal: J Healthc Eng.

# Effect of Eye Movement Training on Sleep Quality of Patients with Advanced Lung Cancer Based on Pittsburgh Sleep Quality Index

**DOI:** 10.1155/2021/9811980

**Published:** 2021-12-16

**Authors:** Haiping Hu, Wenying Yang, Zhimin Liu, Xiaona Zhang, Junmei Shi, Huixia Xu

**Affiliations:** ^1^Department of Oncology, The Fourth Hospital of Hebei Medical University, Hebei Cancer Hospital, Shijiazhuang 050011, Hebei, China; ^2^Department of Blood Purification Center, Wuhan No. 1 Hospital, Wuhan Hospital of Traditional Chinese and Western Medicine, Wuhan 430022, Hubei, China

## Abstract

**Objective:**

To explore the effect of eye movement training on sleep quality of patients with advanced lung cancer based on the Pittsburgh Sleep Quality Index (PSQI).

**Methods:**

120 advanced lung cancer patients admitted to our hospital from January 2019 to January 2020 were selected as the research object and divided into group A (PSQI scores ≥ 10 points, *n* = 60) and group B (PSQI < 10 points, *n* = 60). Routine nursing was performed to both groups, and patients in group A received the eye movement training additionally, so as to compare their PSQI scores, negative emotion scores, adverse reaction rate (ARR), Cancer Coping Modes Questionnaire (CCMQ) scores, and pain scores.

**Results:**

After training, group A obtained significantly better sleep quality (*P* < 0.05), lower negative emotion scores (*P* < 0.001), lower ARR (*P* < 0.05), better CCMQ scores (*P* < 0.05), and lower pain scores (*P* < 0.001) than group B.

**Conclusion:**

Eye movement training should be promoted in practice because it can reduce negative emotions, alleviate pain sensation, improve sleep quality and body condition, and lower the ARR for advanced lung cancer patients.

## 1. Introduction

Lung cancer is a common clinical condition. The latest annual report from the National Cancer Registry in 2018 showed that lung cancer is the malignant tumor with the highest incidence (11.6%) and mortality (18.4%) globally [1]. The causing factors include the environment, pulmonary history, and gene. Lung cancer patients usually present with cough, phlegm, and other clinical symptoms, and some patients even experience the phenomenon of coughing up blood and hoarseness, which greatly affect their life health in a negative way [2, 3]. In the middle to late stage of lung cancer, patients will feel intense cancerous pain that not only affects body condition but also aggravates psychological stress, hence increasing the possibility of sleep disorders. Sleep science is an emerging borderline science, and there are few theoretical studies on this discipline in China currently, not to mention its application, but the relationship between sleep science and cancer has been confirmed by many literatures [4–7]. As patients with advanced lung cancer suffer from various symptoms, more emphasis is placed on treating their somatic symptoms in the clinic with assignment-oriented nursing. Even though some nursing plans add the content of psychological care, it is not targeted enough in managing sleep disorders, so the sleep condition is not well-improved yet [8–10]. With the increasing focus on cancer patients, there are more and more reports involving the quality of life in advanced lung cancer patients, but studies related to their sleep quality are extremely rare. In recent years, it has been reported that oculomotor training can ameliorate the condition of patients with diabetic retinopathy and improve their sleep quality [11], so such intervention measure may also be applied to cancer patients. To explore the effect of eye movement training on the sleep quality of advanced lung cancer patients based on PSQI, 120 patients with advanced lung cancer admitted to our hospital from January 2019 to January 2020 were selected as the research object for the study, with the results summarized as follows.

The article "Effect of Eye Movement Training on Sleep Quality of Patients with Advanced Lung Cancer Based on Pittsburgh Sleep Quality Index" was published in 2021. Journal: J Healthc Eng.

## 2. Materials and Methods

### 2.1. General Information

120 advanced lung cancer patients treated in our hospital from January 2019 to January 2020 were selected as the research object and divided into group A (PSQI scores ≥ 10 points, *n* = 60) and group B (PSQI scores < 10 points, *n* = 60), with no statistical difference in their general information (*P* > 0.05), see Table 1. The study was approved by the Hospital Ethics Committee.

### 2.2. Inclusion Criteria

The inclusion criteria of the study were as follows. (1) The patients or their family members fully understood the study process and signed the informed consent; (2) the patients met the diagnosis criteria for advanced lung cancer after examination [12] and were accepting treatment in our hospital without chemotherapy yet; (3) the estimated survival time of the patients was more than 3 months; and (4) the patients had sleep disorders [13].

### 2.3. Exclusion Criteria

The exclusion criteria for the patients of the study were as follows. (1) Presence of mental problems or inability to communicate with others; (2) suffering from other organic diseases [14]; (3) having the need for analgesic drugs [15]; (4) with sleep disorders not caused by cancer.

### 2.4. Methods

Both groups accepted the routine nursing with the following specific steps. (1) The nursing personnel provided medication intervention and recorded the drug usage according to medical advice. (2) The nursing personnel customized a healthy diet for the patients according to their actual situation and asked their sport preference to guide them to do exercise reasonably. (3) The nursing personnel carried out health education to the patients according to their actual situation, informed the patients and their family members of correct home nursing methods, and adjusted the nursing plan at any time based on the patients' condition, so as to improve the effect and quality of nursing.

The article "Effect of Eye Movement Training on Sleep Quality of Patients with Advanced Lung Cancer Based on Pittsburgh Sleep Quality Index" was published in 2021. Journal: J Healthc Eng.

Eye movement training was given to patients in group A additionally, with the following specific steps. (1) The nursing personnel informed the patients of the function of eye movement training to gain their trust and increase their compliance. (2) The patients were kept in a quiet and relaxed condition, gazed with both eyes into the distance horizontally for 0.5 h, during which the eyeballs were moved inwards (with medial rectus), upwards/inwards (with superior rectus), downwards/inwards (with inferior rectus), upwards/outwards (with inferior oblique), and downwards/outwards (with superior oblique) for 36 times each and moved annular from left to right to the maximum extent. (3) The patients did the eye movement training once a day and 5 days a week for 1 month. (4) The sleep index table was put at the foot of the patients' beds for dynamic observation; their sleep indexes were evaluated daily during training, and outpatient evaluation and guidance were provided at the time of discharge from the hospital.

### 2.5. Observation Criteria

1. Pittsburgh Sleep Quality Index (PSQI): six factors in the PSQI scale (sleep quality, sleep latency, sleep efficiency, use of sleeping medication, and daytime dysfunction) were selected and compared before and after training. The total score was 18 points, with 0–3 points for each item, and lower scores indicated better sleep [16].
2. Negative emotion scores: the negative emotions were evaluated by the Self-Rating Anxiety Scale (SAS) and Self-Rating Depression Scale (SDS) before and after training, and each scale contained 20 items and has a total score of 100 points. Higher scores indicated that the negative emotions of patients were more serious [17].
3. Adverse reaction rate (ARR): the adverse reactions included digestive tract reaction, allergic reaction, injury of skin and mucous, and myelosuppression, and the number of patients with adverse reactions was counted.
4. Cancer Coping Modes Questionnaire (CCMQ): it included 26 items and 5 dimensions, of which the higher scores on confrontation and avoidance and depression indicated a more positive attitude towards the condition, while the higher scores on acceptance-resignation, imagination, and abreaction indicated a more negative attitude towards the condition [18].
5. Pain scores: the Chinese version of the Brief Pain Inventory (BPI-C) scale was used to evaluate the pain degree of patients in both groups before and after training, which covered five dimensions such as the most serious pain to the slightest pain within 24 hours. On a scale of 0–10 points, higher scores indicated more serious pain [19].

The article "Effect of Eye Movement Training on Sleep Quality of Patients with Advanced Lung Cancer Based on Pittsburgh Sleep Quality Index" was published in 2021. Journal: J Healthc Eng.

### 2.6. Statistical Processing

In this study, the data processing software was SPSS20.0, the picture drawing software was GraphPad Prism 7 (GraphPad Software, San Diego, USA), items included were enumeration data and measurement data, methods used were *X*^2^ test and *t*-test, and differences were considered statistically significant at *P* < 0.05.

## 3. Results

### 3.1. Comparison of PSQI Scores

After training, the sleep quality of group A was significantly better than that of group B (*P* < 0.05), see Table 2.

### 3.2. Comparison of Negative Emotion Scores

After training, the negative emotion scores of group A were significantly lower than those of group B (*P* < 0.001), see Table 3.

### 3.3. Comparison of ARR

The ARR of group A was significantly lower than that of group B (*P* < 0.05), see Figure 1.

Note: in Figure 1, the black areas indicate digestive tract reaction, the dark gray areas indicate allergic reaction, the light gray areas indicate injury of skin and mucous, and the white areas indicate myelosuppression; the left image indicates group A, and the right image indicates group B.

The number of patients with digestive tract reaction in group A and group B was 30 and 40, respectively (*X*^2^ = 11.868, *P* < 0.05).

The number of patients with allergic reaction in group A and group B was 24 and 36, respectively (*X*^2^ = 4.800, *P* < 0.05).

The number of patients with injury of skin and mucous in group A and group B was 24 and 42, respectively (*X*^2^ = 10.909, *P* < 0.05).

The number of patients with myelosuppression in group A and group B was 25 and 45, respectively (*X*^2^ = 13.714, *P* < 0.05).

### 3.4. Comparison of CCMQ Scores

After training, the CCMQ scores of group A were significantly better than those of group B (*P* < 0.05), see Table 4.

### 3.5. Comparison of Pain Scores

After training, the pain scores of group A were significantly lower than those of group B (*P* < 0.001), see Figure 2.

Note: in Figure 2, the horizontal axis indicates before and after training, and the vertical axis indicates the pain scores (points); the black areas indicate group A, and the gray areas indicate group B; and *∗* indicates *P* < 0.001.

The data before training indicated that the results of comparing the pain scores between group A and group B were not statistically different (4.98 ± 0.54 vs 4.87 ± 0.58, *P* > 0.001).

The article "Effect of Eye Movement Training on Sleep Quality of Patients with Advanced Lung Cancer Based on Pittsburgh Sleep Quality Index" was published in 2021. Journal: J Healthc Eng.

The data after training indicated that the pain scores of group A were significantly lower than those of group B (3.65 ± 0.35 vs 4.25 ± 0.48, *P* < 0.001).

## 4. Discussion

At present, the number of patients suffering from malignant tumors is increasing year by year worldwide, expanding the group of cancer patients continuously. Reports indicated that there are more than 2 million new lung cancer patients every year with poor prognosis. The academia has gradually recognized that the purpose of treating cancer is not only limited to resection of tumors but also to improve the life health of patients and their quality of life. Lung cancer is one of the most common cancers in China, and 47% of lung cancer patients experience sleep disorders [20] that seriously compromise the treatment efficacy. Patients present severe nausea and decreased appetite from long-term treatment and cancer-induced fatigue after progressing to the end stage of the disease; at this time, their depression is more pronounced and their sleep quality decreases even further, raising the possibility of sleep disorders to over 50%. As sleep quality is closely related to life quality and treatment effect, and clinical practice has regarded life quality as one of the first indicators to evaluate the prognosis of patients, it is crucial to increase the efforts in conducting corresponding research.

Sleep science is an emerging science in China, but it is not well studied in academia at present nor fully applied in practice, so there is still a lack of well-established measures for sleep quality improvement in China. The oculomotor training selected in this study is often used in the treatment of diseases such as cognitive impairment. As an aerobic exercise of the brain, it is able to improve the cognitive ability of patients and reduce their physical and mental burden, and Secinti et al. stated that oculomotor training can help the body of patients to enter a state of complete relaxation, hence it is positive in weakening the anxiety of patients [21]. The study showed that the negative emotion scores after training of group A were significantly lower than those of group B (*P* < 0.001), indicating that the oculomotor training successfully brought the patients into a quiet and relaxed atmosphere to enable them to take control of themselves again, greatly improve their self-efficacy, and alleviate their anxiety. Since anxiety and depression are the major factors that trigger sleep disorders in advanced lung cancer patients [22], the sleep quality will be improved with these emotions alleviated, as indicated by shorter sleep latency and lower likelihood of using sleep medication.

The article "Effect of Eye Movement Training on Sleep Quality of Patients with Advanced Lung Cancer Based on Pittsburgh Sleep Quality Index" was published in 2021. Journal: J Healthc Eng.

It is indisputable that sleep quality is of positive relevance with life health [23]. For instance, the study by Pongthavornkamol et al. showed that high-quality sleep can improve the psychological and body state and accelerate the rehabilitation progress, hence it is in favor of body recovery [24], while poor sleep quality affects the regular work and rest, disrupts the circadian rhythm, and negatively influences the quality of life and treatment effect of patients. Better sleep quality will improve the physical and psychological conditions in patients. Therefore, group A obtained significantly better CCMQ scores (*P* < 0.05) and lower pain scores (*P* < 0.001) than group B after training, indicating that because of a good sleep, patients in group A promoted their self-awareness, greatly enhanced their confidence in treatment, kept a more positive mind, and improved their body tolerance and that the sleep quality can affect the prognosis of advanced lung cancer patients.

In addition, the study also concluded that the ARR of group A was remarkably lower than that of group B (*P* < 0.05), which was consistent with the findings of Kizilgz and other scholars. In their study, patients in the experimental group received routine nursing combined with eye movement treatment, and patients in the control group were given the routine nursing only, and it was concluded that after treatment, the probabilities of patients in the experimental group having digestive tract reaction, allergic reaction, injury of the skin, and mucous and myelosuppression were 48%, 50%, 48% and 45%, respectively, which were obviously lower than those in the control group (*P* < 0.05) [25], indicating that the eye movement training could promote the body status by improving the sleep quality, thereby enhancing the tolerance and lowering the possibility of adverse reactions in patients.

In conclusion, eye movement training should be promoted in practice because it can reduce negative emotions, alleviate pain sensation, improve sleep quality and body condition, and lower the ARR for advanced lung cancer patients.

## Figures and Tables

**Figure 1:** Comparison of ARR. (a) Group A = 103. (b) Group B = 171.

**Figure 2:** Comparison of pain scores before and after training ($\bar{x}$ ± *s*, points).

**Table 1:** Comparison of general information.

Group	Group A (*n* = 60)	Group B (*n* = 60)	*X* ^2^/*t*	*P* value
Gender			0.034	0.853
Male	35	34		
Female	25	26		
Age (years old)				
Range	32–74	33–74		
Mean age	61.21 ± 6.20	61.23 ± 6.21	0.018	0.986
TNM stage			0.034	0.854
IIIb	34	33		
IV	26	27		
Distant metastasis				
Lymphatic metastasis	30	30	0.000	1.000
Bone metastasis	16	17	0.042	0.838
Liver metastasis	10	11	0.058	0.810
Metastasis to other parts	4	3	0.152	0.697
Clinical history				
Diabetes	8	9	0.069	0.793
Hypertension	12	13	0.051	0.822
Coronary heart disease	7	6	0.086	0.769
Lung disease	10	11	0.058	0.810
Educational level				
Junior high school and below	12	13	0.051	0.822
Senior high school	30	30	0.000	1.000
College and above	18	17	0.040	0.841
Monthly income (yuan)			0.035	0.852
≥3000	36	37		
<3000	24	23		

The article "Effect of Eye Movement Training on Sleep Quality of Patients with Advanced Lung Cancer Based on Pittsburgh Sleep Quality Index" was published in 2021. Journal: J Healthc Eng.

**Table 2:** Comparison of PSQI scores after training ($\bar{x}$ ± *s*, points).

Group	Sleep latency	Sleep duration	Sleep efficiency	Sleep disorders	Use of sleeping medication	Daily dysfunction	Sleep quality
Group A	1.68 ± 0.65	1.18 ± 0.24	0.59 ± 0.35	1.00 ± 0.32	1.02 ± 0.24	1.45 ± 0.65	1.75 ± 0.65
Group B	2.01 ± 0.54	1.52 ± 0.28	1.20 ± 0.39	1.23 ± 0.65	1.38 ± 0.34	2.10 ± 0.54	2.00 ± 0.54
*t*	3.025	7.141	9.017	2.459	6.700	5.958	2.292
*P* value	0.003	0.000	0.000	0.015	0.000	0.000	0.024

**Table 3:** Comparison of negative emotion scores ($\bar{x}$ ± *s*, points).

Group	SDS before and after		SAS before and after	
Group A	58.65 ± 6.68	42.11 ± 5.98	60.11 ± 10.65	40.65 ± 5.68
Group B	58.84 ± 6.57	48.98 ± 6.95	61.20 ± 10.54	47.11 ± 5.65
*t*	0.157	5.804	0.563	6.246
*P* value	0.876	0.000	0.574	0.000

**Table 4:** Comparison of CCMQ scores after training ($\bar{x}$ ± *s*, points).

Group	Confrontation	Avoidance and depression	Acceptance-resignation	Imagination	Abreaction
Group A	3.25 ± 0.54	1.68 ± 0.65	2.18 ± 0.34	1.45 ± 0.25	1.54 ± 0.54
Group B	2.54 ± 0.65	2.20 ± 0.48	2.65 ± 0.54	1.87 ± 0.60	1.89 ± 0.68
*t*	6.508	4.985	5.705	5.005	3.122
*P* value	0.000	0.000	0.000	0.000	0.002

## Data Availability

Data that supported the findings of this study are available on reasonable request from the corresponding author.
